RETRACTED

# Lead Exposure Induced Neural Stem Cells Death via Notch Signaling Pathway and Gut-Brain Axis

**DOI:** 10.1155/2022/7676872

**Published:** 2022-10-04

**Authors:** Lijuan Sun, Yuankang Zou, Peng Su, Chong Xue, Diya Wang, Fang Zhao, Wenjing Luo, Jianbin Zhang

**Affiliations:** ^1^Department of Occupational and Environmental Health, The Ministry of Education Key Lab of Hazard Assessment and Control in Special Operational Environment, School of Public Health, Fourth Military Medical University, No. 169 Chang Le West Rd., Xi'an, Shaanxi 710032, China; ^2^Key Laboratory of Resource Biology and Biotechnology in Western China, Ministry of Education, School of Medicine, Northwest University, 229 Taibai North Road, Xi'an 710069, China

## Abstract

Numerous studies have examined the effects of lead (Pb) on cognitive ability. It is essential for the brain to maintain its functions through the differentiation of neural stem cells into various types of cells. Despite this, it remains unclear how Pb exposure affects neural stem cells and how it does, so the Pb-exposed mice were treated with the Notch inhibitor DAPT after we established the Pb exposure models. Neuronal stem cells and autophagy were assessed by immunofluorescence staining and western blot. The microbiota of the feces was also analyzed using the 16S rRNA amplicon sequencing technique. In this study, we found that Pb exposure caused neural injuries and deficits in neural stem cells, whereas DAPT rescued the damage. With DAPT, Pb-induced autophagy was partially reversed. Exposure to Pb also reduced inflammation and damaged gut barrier function. Furthermore, Pb exposure led to low bacterial diversity, an increase in pathogen abundance, and an unusual mode of interaction. Taken together, this study revealed that damages in neural stem cells contributed largely to cognitive impairment during Pb exposure, and this process was partially dependent on the Notch pathway and gut dysbiosis.

## 1. Introduction

As one of the most widely known heavy metals, lead (Pb) is recognized as an important pollution source for air, water, and soil. In addition to damage problems in the nervous system, Pb also cause problems in cardiovascular system, hematological system, and kidneys. Pb exposure has a great impact on cognitive and behavioral development. Accumulating studies showed that Pb exposure increases the risk of major depressive disorder, anxiety disorder, and panic disorder [1]. The workers exposed to Pb often showed impaired attention, speed, working memory, visuospatial abilities, and general intellectual performance. Childhood with high Pb exposure level are at higher risk of lower Intelligence Quotient (IQ) scores and higher risk of behavior problems, including hyperactivity, inattention, and antisocial behavior [2]. More importantly, it was also found that Pb exposure during childhood is linked with long-term negative effects on psychological well-being and personality in adulthood [3, 4]. Pb exposure in the environment continues to be a serious public health problem.

RETRACTED

Stem cells are neuronal precursors that differentiate into various types of cells, including neurons, oligodendrocytes and astrocytes. In the event that this homeostasis is disrupted, numerous defects can appear, such as defects in nervous system development, motor disturbance, and cognitive symptoms. As previously reported, in zebrafish, Pb exposure caused impaired neurogenesis and abnormal apoptosis in the neuronal cells. In a rat model exposed to Pb, it was reported that the neuronal stem cells are less likely to survive and proliferate. Furthermore, Pb is also shown to reduce the proliferation and viability of the neuronal progenitor cells [5].

Development and patterning of neuron stem cells are controlled by a complex regulatory network, which is affected by various signaling pathways, including Notch, Wnt signaling, and receptor tyrosine kinase. They affect the determination of cell fate.

Notch signaling is crucial for brain development, not only for stem cell proliferation but also for neuronal differentiation, and for keeping neural precursors undifferentiated and inhibiting neural differentiation. However, despite stem cells and Notch pathways playing key roles in the nervous system, their cross-talk and roles in Pb exposure-induced cognitive deficit remain largely unexplored.

Accumulating evidence from human and animal studies suggests that environmental pollutants can alter gut microbiota, disrupting physiological homeostasis, partly contributing to the development of nervous system diseases. The commensal bacteria are sensitive to heavy metals. Cadmium can cause gut damage and dysbiosis, and some recent studies showed that Pb exposure also affects the digestive system and intestinal microbiota in birds. Furthermore, probiotics (*Bacillus coagulans* R11) are considered useful tools for removing lead ions from the gut and protecting the gut against damage due to villitis [6]. It has been reported that Notch signaling can regulate the differentiation of secretory cells and absorptive cells in the gut, which may shape the composition of mucus-associated bacteria [7].

In this research work, the effect of Pb exposure on cognitive ability in mice was investigated. Subsequently, it was explored whether Notch signaling is involved in this process. This study demonstrated that the Notch pathway in vivo regulated the neural stem cells. It was also discovered that Pb induces elevated autophagy and this process can be restored by DAPT. Additionally, this study shed light on the peripheral factors that contribute to the negative effects of Pb exposure on cognitive performance, and may provide clues as to how Pb-related cognitive impairments may be treated.

RETRACTED

## 2. Materials and Methods

### 2.1. Ethics Statement

A committee of the Institute of the Fourth Military Medical University approved this study (No. IACUC-20190950) and throughout all experiments involving animals, the National Institutes of Health Guide for the Care and Use of Laboratory Animals was followed.

### 2.2. Animals

These studies utilized mice aged 3 weeks (C57BL/6). The mice were kept in a temperature-controlled environment (22°C). On day 3, each of the mice were randomly assigned to one groups, including the control group, the low-dose Pb group, and the high-dose Pb group. In deionized water, Pb acetate was dissolved at various concentrations (0, 100 ppm, and 300 ppm). Model was constructed using the drinking water method and the three group-control, low-dose Pb exposure group, and high-dose Pb exposure group-were given deionized water that contained lead acetate. The exposure lasted for eight weeks. Additionally, all mice in the three groups were always provided with food. After 8 weeks of exposure to Pb, behavioral tests were conducted. In accordance with the “Guide for the Care and Use of Laboratory Animals of the National Institute of Health”, the study was conducted.

### 2.3. Pb Concentration Analysis

The left ventricles of mice were used for collecting blood samples (600 *μ*l) for analysis of Pb levels in the blood. Measurements of Pb levels were carried out by a graphic furnace and an atomic absorption spectrometer (AAS).

### 2.4. Morris Water Maze

The test was performed as previously reported [8]. Our experiments were conducted in a tank containing opacified water of 120 cm diameter and 50 cm depth. An above-water video camera monitored the mice from a platform with a diameter of 10 cm. The trial involved placing a mouse in the water at one starting point. Animals that had difficulty finding the platform within two minutes were guided to it, where they stayed for 10 seconds. A 120-second swim was allowed after the hidden platform test without any restrictions on the mice. Swim speed, escape latency, and distance traveled were measured during each trial. Each quadrant's entries, swimming speed, and time were recorded with cameras. In order to analyze these data, we used Noldus Ethovision XT (Wageningen, Netherlands).

### 2.5. Cue and Contextual Fear Conditioning

The test was conducted using the NIR Video Fear Conditioning System for mice (Med Associates, Inc., St. Albans, VT, USA). After a 2-min exploration time, we performed two pairs of conditioned-unconditioned stimuli pairings (white noise, foot shock intensity, duration of 30 seconds, and foot-shock intensity). 24 hours after the training, we conducted context tests. After six minutes of training, we conducted cue tests in a separate room one hour later. In the contextual, precued and cued tests, we scored the animals every 10 seconds whether they were frozen or not.

RETRACTED

### 2.6. Western Blot

We analyzed total proteins from colon tissues using SDS-PAGE, and then we incubated the membrane with antibodies against ZO-1 (ThermoFisher, 1: 1000); ZO-2 (Cell Signaling Technology, #2847, 1: 1000); E-cadherin (BD Biosciences, 1 : 1000); Occludin (ThermoFisher, 1 : 1000); Claudin 3 (ThermoFisher, 1 : 1000); Beclin1 (Cell Signaling Technology, #3738, 1 : 1000); LC3 (Cell Signaling Technology, #3868, 1 : 1000); Atg 5 (CST, #12994, 1 : 1000); Notch1 (Abcam, ab52627, 1 : 1000); RBP-J (Abcam, ab180588, 1 : 1000); Hes1 (Abcam, ab119776, 1 : 1000); Hes2 (Abcam, ab168071, 1 : 1000); mTOR (CST, #2972, 1 : 1000); p-mTOR (CST, #5536, 1 : 1000); P70s6k (CST, #9202, 1 : 1000); p-P70s6k (CST, #97596, 1 : 1000) and *β*-actin. After overnight at 4°C, they were incubated with the secondary antibodies (anti-rabbit or anti-rat) for 1 h at 25°C. Then the images were captured.

### 2.7. Immunofluorescence

Blocking the slides with 3% BSA, 0.2% TWEEN 20 in PBS, incubating them with primary antibodies against ZO-2 (Cell Signaling Technology, 1 : 100) overnight, and then secondary antibodies (Servicebio, 1 : 300) for 1 h.

### 2.8. 16S rDNA Sequencing and Analysis

Stool DNA Kits were used to extract fecal genomic DNA from the pellets (Omega Bio-tek, Inc., Norcross, GA, USA). We used primers F1 and R2 (5′-CCTACGGGNGGCWGCAG-3′ and 5′-GACTACHVGGGTATCTAATCC-3′) located in 16S rRNA gene 341–805 of Escherichia coli for amplifying the V3–V4 regions of the sample. The sequencing library was constructed and paired-end reads were generated on a MiSeq platform, as the manufacturer's instructions. FASTQ software was used for merging and filtering the sequencing data. Diversity indices were calculated by QIIME2. A network analysis was conducted by bacterial genera. We calculated Spearman rank correlations, and if the Spearman rank correlation coefficient was greater than 0.8 and a significance of *P* < 0.05, we considered that to be a robust correlation. Gephi software was used to construct correlation networks with robust correlations.

### 2.9. Statistical Analysis

Data for behavioral tests were presented in the form of means and standard errors of the means. Comparing two groups was done using *t*-tests of the students. We used the *R* package vegan to analyze the bioinformatics data of gut microbiota. Significant levels were set at *P* < 0.05.

RETRACTED

## 3. Results

### 3.1. Exposure to Pb Caused Significant Cognitive Impairment in Mice

The cognitive ability was examined by two independent behavioral tests, i.e. Morris water maze tests and fear condition box tests, as the protocol shown in Figure 1(a). The serum Pb concentration of the mice in the Pb exposure groups were higher than that of the control group, *P* < 0.05 and *P* < 0.01, respectively, reflecting a sufficient Pb exposure, Figure 1(b). Fear condition box test showed that the freezing time in the two Pb exposure groups was lower, both in context and conditioning stimulus, *P* < 0.05, implying impaired environmental memory, Figure 1(c). In the Morris water maze test, no influence on swimming speed after Pb exposure was recorded, however, the platform and edge frequencies in the two Pb groups were decreased, and at the fifth day of training, the significant difference was observed, *P* < 0.05, Figure 1(d). These data showed that mice exposed to Pb developed significant environment-dependent and spatial-dependent memory problems.

### 3.2. Pb Exposure Reduced Neuron Stem Cells and Regulated Autophagy in the Dentate Gyrus

In the brain, the neural stem cells produce new neurons that contribute to complex sensory and cognitive functions. To investigate the potential mechanisms of how Pb exposure regulates cognitive function, 5-bromo-2′-dexoyuridine (BrdU) staining with fluorescence was performed to label cell proliferation from the control and high dose-Pb exposure group. The control and Pb groups were observed to have markedly different BrdU(+) cells. The mice in the Pb group had fewer BrdU(+) cells in the dentate gyrus (DG) (Figure 2(a)). SOX2 is an important transcription factor of mediating cell fate specification in the human neural progenitor cells [9], playing a key role in various phases of cell fate and differentiation. The expression level of SOX2 was analyzed and it was found that the SOX2(+) cells sharply reduced in the Pb exposure group (Figure 2(b)). These results imply that after Pb exposure, the number of neural stem cells significantly decreases.

In addition to being an essential cell survival mechanism, the autophagy is an essential lysosome-dependent catabolic process involved in normal development and physiology [10]. To determine whether autophagy is responsible for neurogenesis decline caused by Pb exposure, LC3II staining with fluorescence showed that Pb had induced increased autophagy in the dentate gyrus, as shown in Figure 2(c). Autophagy flux was found to have increased in the Pb exposure group, Figure 2(d). It was also found that the expression levels of Beclin 1, LC3I, and LC3II increased after Pb exposure. Based on these results, the dentate gyrus demonstrated an elevated autophagy flux after Pb exposure.

RETRACTED

### 3.3. Suppression of Cognitive Deficits Induced by Pb Exposure Is Prevented by Inhibition of Notch Signaling

In mammals, Notch pathways play an essential role in determining cell fate [11]. To explore the regulatory mechanism of Pb exposure on cognitive deficits, the expression level of Notch1, RBP-J, Hes1, and Hes2 was assessed by western blotting. The results showed that the expressions of Notch1, RBP-J, Hes1, and Hes2 in the dentate gyrus and olfactory bulb were significantly increased when treated with Pb exposure (*P* < 0.05), as shown in Figures 3(a) and 3(b). To determine the role of the Notch signaling pathway in Pb exposure-related cognitive deficits, the effect of inhibitor of Notch1 on Pb exposure was assessed. Notch1-expressing in the Pb + DAPT group showed no significant differences compared to that of the Pb group. There was, however, a decreased level of expression of the downstream effector of Notch signals, which affects neuronal progenitor fate decisions. Several genes related to neuronal differentiation were decreased, such as RBP-J, Hes1, and Hes2, *P* < 0.05, as shown in Figure 3(c). From here on, the Notch signaling pathway can be referred to have been involved in the Pb exposure-related cognitive deficits. Consistent with these findings, DAPT also prevented the Pb exposure-related cognitive deficits. As shown in Figure 3(d), the freezing time of the mice in the Pb + DAPT group was largely higher than that in the Pb group, including in the context and conditioning stimulus conditions. Correspondingly, as to the Morris water maze test, there was no difference in swimming speed for the four groups, but the platform+ edge frequency of the mice in the Pb + DAPT group increased as compared with that in the Pb group, on the fifth day of training, a significant change took place, *P* < 0.05. Altogether, it was identified that Pb exposure could impair cognitive ability through the Notch signaling pathway.

### 3.4. The Protective Effects of Notch Inhibition on Cognitive Deficits Depend on Autophagy

Recently data has shown that axon injury can activate autophagy by limiting Notch signaling [12]. In this study, the data also showed that Pb exposure activated autophagy in the dentate gyrus region. These findings lead us to verify that the protective effects of Notch inhibition on cognitive deficits depend on autophagy. Autophagy flux levels in the Control, Pb, DAPT, and Pb + DAPT groups were examined by western blot, and the results showed that the expressions of Beclin1, Atg5, and LC3I were significantly decreased in the Pb + DAPT group when compared with that in the Pb group, *P* < 0.05, but the expression of LC3II showed no significant alteration, as shown in Figure 4(a).

RETRACTED

There are a number of sequential events that occur during autophagy, including initiation, elongation, nucleation, recruitment of cargo, and maturation of the autophagosome, transit, and degradation [13]. These events are critically coordinated by an intricate network. The mammalian target of rapamycin (mTOR) is regarded as a master regulator of autophagy [14]. To further study the potential mechanism of autophagy regulation in Pb exposure, the expression level of the mTOR pathway was evaluated, as shown in Figure 4(b). Pb exposure induced remarkably decreased p-mTOR and p-P70s6k, and DAPT partially recovered the shift, as shown in Figure 4(b). These results together indicate that Notch inhibition rescued Pb exposure-related cognitive deficits partly through the mTOR/autophagy pathway.

### 3.5. Pb Exposure Induced a Low Inflammatory Response in the Gut and Gut Dysbiosis in Mice

Recent preclinical and clinical studies have shown bidirectional interaction within the gut-brain axis. The gut exerts the brain through the gut microbiota metabolites, microbiota-derived products, and gut hormones [15]. In light of these findings, we decided to investigate whether Pb exposure lead to altered intestinal philosophy. This study found that Pb exposure increased higher gut permeability, and the expression levels of several markers of gut tight junctions were significantly decreased, such as E-cadherin, Claudin-3, ZO-2, and ZO-1, *P* < 0.05, as shown in Figure 5(a). In line with these findings, in the Pb exposure group, hematoxylin-eosin staining of the colon and jejunum showed sparsity of intestinal villus and edema, and an enhanced inflammation cells infiltration, as shown in Figure 5(b) and 5(c), implying a low inflammatory response of the gut after Pb exposure. The gut exerts various effects on the brain through gut microbiota. Subsequently, in order to measure gut microbiota composition, 16 s rRNA genes were sequenced. We found that the Shannon diversity index was significantly decreased in two Pb exposure groups, as shown in Figure 5(d). Similarly, the Principle Coordinates Analysis (PCoA) plots of Bray-Curtis dissimilarity showed that the dots of the two Pb exposure groups were distinct from those of the control group. It is worth noting that the dots of the high-dose Pb exposure groups were farther away from that of the control group, as shown in Figure 5(e). These results suggest that Pb exposure leads to gut injury and dysbiosis.

RETRACTED

### 3.6. Pb-Exposure Induced Gut Dysbiosis Is Tightly Associated with Cognitive Deficits in Mice

A network comprising all the bacterial genera in each of the three groups at the genus level was constructed to examine the modulatory effect of Pb exposure on gut microbiota, which showed that Pb exposure led to more complicated networks, i.e. V/E = 76/241 in low dose group and V/E = 108/1478 in high dose group, when compared with the control group, i.e. V/E = 68/145. Most specifically, in the high dose exposure group, the interaction mode was remarkably different from that of the other two groups, as shown in Figure 6(a). The most complicated network in the high-dose group is more likely to have a foundation guild to affect the host phenotypes.

To evaluate the specific bacteria that were affected by Pb exposure, this study selected the bacterial taxon with different abundance among the three groups. The abundance of Bacteroides, Lactobacillus, Escherichia/Shigella, Clostridium XIVb, and Roseburia significantly and consistently increased in the two Pb exposure groups. In addition, the abundance of Alloprevotella, Parabacteroides, Saccharibacteria_ genera_incertae_sedis, Prevotella, Ruminococcus, Clostridium IV, Butyricicoccus, Eubacterium, and Intestinimonas decreased following low dose and high dose Pb exposure. The linear discriminant analysis of effect size (Lefse) showed that in the Pb exposure group, a higher abundance of bacteria taxon primarily originated from Deferribacteres phylum, Gammaproteobacteria class, Erysipelotrichia class, and Bacilli class. The bacteria taxon with low abundance in the Pb exposure group primarily originated from Tenericutes phylum, as shown in Figure 6(c). The relationship analysis showed that the expressions of Escherichia/Shigella, proteus, Bacteroides, Clostridium_XVIII, Lactococcu, Veillonella, Roseburia, and Gemella are contrary with most intestinal bacteria.

To identify correlations between the altered bacteria and behavioral parameters, an association analysis was performed. It was found that most of the shifted gut microbiota were significantly related to the level of serum Pb and cognitive behavior index, as shown in Figure 6(d). Taken together, these results suggest that Pb exposure-related gut dysbiosis may contribute partially to the cognitive deficits.

## 4. Discussion

The problem of heavy metal pollution has become a major concern all over the world. Evidence demonstrates that Pb exposure causes cognitive impairment in certain individuals. However, there is a limited intervention to protect the deficits related to Pb exposure. In this study, it was observed that the Pb exposure-induced cognitive deficits can be partially restored by Notch inhibitor DAPT, and its effect is dependent on the mTOR/autophagy axis. Additionally, it was found that gut dysbiosis may also contribute to the Pb exposure-related behavior alteration.

RETRACTED

Prior work suggested that Pb exposure can result in significant decline in cognitive and memory abilities [3, 4, 16]. As previously described, this study also found an impaired cognitive ability, confirming the successful establishment of the Pb exposure model. Pb can impair nervous system by several ways: aptosis, autophagy, and inflammatory reaction, all of which can induce nervous system disorders and neuron impairment. There are certain amount of neural stem cells remained in hippocampal DG region of adult mice. These neural stem cells play important roles in the maintenance of nervous system function. Neuron injury was detected in our lead exposure experiments. In our further studies, a decreased number of neuron was observed in hippocampal DG region, indicating lead exposure may influence the survival of neural stem cells. Neural stem cell is the most primitive state of other types of differentiated cells. Therefore, we paid attention mainly to neural stem cells. Maintenance of the neural stem cells pool after various stresses is essential for preventing impairment of neurogenesis. Heavy metal pollution may negatively impact adult neurogenesis via the decrease in adult neurogenesis. This study focused on the neuron stem cells alteration in the DG region as it plays a vital role in hippocampus-dependent memory function. This study's data showed that Pb exposure had reduced neuron stem cells verified by BrdU and SOX2 staining in the DG region. This is an important complement for the explanation of Pb exposure-related cognitive deficits, which has not been investigated so far.

The fact that Notch signaling is a key regulator for the neuronal progenitor proliferation and neuronal differentiation urges us to verify the contributions of Notch in the abnormal neuron stem cells. Through expression analysis and inhibition intervention, this study found evidence that Notch signaling plays a key role in the neurological phenotypes during Pb exposure. Accordingly, the protection offered by Notch inhibitor DAPT is most possibly related to the recovery of neuron stem cells. Also, to our knowledge, this is the first attempt for the Notch inhibitor to restore the cognitive impairment during Pb exposure. This may also provide a promising intervention choice for Pb exposure-related cognitive deficits.

RETRACTED

It is increasingly recognized that abnormal autophagy pathways can contribute to pathogenesis in AD and PD, as it preserves the complex neuronal architecture of various regions in the brain [17]. This study showed that the autophagy increased after Pb exposure, and Notch inhibition rescued Pb exposure-related cognitive deficits partly through the mTOR/autophagy pathway. As to the interaction between Notch and mTOR signaling pathways, recent research indicates that mTORC1 signaling is reduced when Notch is inhibited in gastric cancer cells, supporting the idea that mTOR is downstream of Notch [18], which is consistent with this study. However, more evidence is needed to fully resolve with regard to the interaction of mTOR and Notch signaling, which for now remains mysterious. The question remains whether the Pb exposure is robustly linked to Notch and mTOR signaling, or the two pathways complicated interaction during the process.

The data in this study showed that DAPT cannot restore all the cognitive deficits, suggesting that the Notch signaling may act partially to the phenotypes. Other factors may also be involved in the responsiveness to Notch. Accumulating evidence showed that although the exact mechanisms have not been fully understood, gut microbiota is known to contribute to brain physiological, behavioral, and cognitive functions [19, 20]. Accordingly, there are also scattered reports of Pb exposure and gut microbiota with smaller duplications. These studies have pointed to Pb exposure-induced gut microbiota disturbance, including altered alpha-diversity, decreased Clostridiales, Ruminococcus, and Oscillospira, although the results from various studies are not consistent [21, 22]. However, no detailed explanation for the possible core bacteria has been established. Thus, in this study, network analysis was performed at the genus level, which highlights the remarkable changes in complicated networks in the high dose group, which is more likely to be a foundation guild to affect the host phenotypes. Furthermore, this microbiota signature may be used as a screening tool for Pb exposure-related neural injury.

Of particular interest is the overgrowth of *Escherichia/Shigella* in the gut microbiota, is thought to involve in the impairment of cognitive ability. Although it has remained elusive how the gut microbiota played their roles in regulating central nervous system functions, it has been accepted that gut permeability plays a key role in immune regulation and cognition [23]. The gut microbiome regulates immune cell populations in part through metabolites and other products, which can regulate systemic immune response via Toll-like receptors among other innate and adaptive immune pathways [24, 25]. *Escherichia/Shigella* is commonly regarded as a pathogenic organism that can trigger gut inflammation [26]. As a result, this study speculates that gut dysbiosis may be related to cognitive impairment in mice although further identification is required.

RETRACTED

Some gut microbiota-derived metabolites play an indispensable role in intestinal stem cell development. For example, lactate derived from the microbiota promotes epithelial development in intestinal stem cells, which is dependent on Wnt/*β*-catenin or Notch signals [27]. Apropos of this, this event may also have been crucial to the neuron stem cells, marking the Pb exposure-related gut dysbiosis involved in the renewal and differentiation of neuronal progenitor cells. A change in the gut microbiota may lead to an increase in neuron production. This may represent a new mechanism to explain cognitive deficits resulting from Pb exposure.

Major strengths are the exploratory attempt of a new compound in this study. Our studies showed that DAPT can partially rescue the cognitive deficits during Pb exposure. Thus, this provided us a potential strategy for Pb exposure. More interestingly, we found a group of gut bacteria whose interaction mode is largely distinct from that of the control group, which implied a foundation guild to affect the host phenotypes. This also provided us a possible explanation for the complication of Pb exposure.

This study possesses several limitations of note. Significant over-activation of autophagy was found in the DG region, and DAPT reliably restored the over-autophagy. These findings acknowledge an important role of the Notch pathway in this process, and this combined with the effects of the Notch inhibitor, makes it difficult to argue for their interaction in the process. Further studies are still needed to clarify their interaction. In addition, although remarkable changes in the gut microbiota were found, it is still not confirmed that the alteration in gut microbiota causes cognitive impairment. In order to understand the accompanying or causal relationships between fecal and intestinal microbiota, transplants of feces are required.

## 5. Conclusion

Based on this study, the neuron stem cell injury through Notch signaling may be considered a new candidate to contribute to the neurological phenotypes during Pb exposure. Meanwhile, the effects of the factors beyond the central nervous system cannot be neglected. In light of this study's findings, there are important implications for understanding neuron stem cells in the face of heavy metal pollution, as well as an alternative design of interventional strategies by targeting Notch for the treatment of the consequences of Pb exposure.

RETRACTED

## Figures and Tables

**Figure 1:** Exposure to Pb caused significant cognitive impairment in mice. (a) Experimental schedule of the present study. (b) Concentration of blood lead in three groups. (c) Freeze time in the context and conditioning stimulus during the cue and contextual fear conditioning test in the three groups. (d) Swimming speed, Platform+Edge frequency, and Lantency period during Morris water maze test in the three groups. ^∗^*P* < 0.05.

**Figure 2:** Pb exposure reduced neuron stem cells and regulated autophagy in dentate gyrus. (a) Representative images of BrdU staining with fluorescence. (b) Representative images of SOX2 staining with fluorescence in the dentate gyrus. (c) Representative images of LC3II staining with fluorescence in the dentate gyrus. (d) Western blot analysis and shading analysis of autophagy related gene. ^∗^*P* < 0.05, ^∗∗^*P* < 0.01.

**Figure 3:** Suppression of cognitive deficits induced by Pb exposure are prevented by inhibition of Notch signaling. (a) Western blot analysis and shading analysis of Notch1, RBP-J, Hes1, and Hes2 in DG in Hippocampus in the three groups. (b) Western blot analysis and shading analysis of Notch1, RBP-J, Hes1, and Hes2 in olfactory bulb in the three groups. (c) Western blot analysis and shading analysis of Notch1, RBP-J, Hes1, and Hes2 in DG in Control, high-dose Pb exposure, DAPT, and high-dose Pb exposure+DAPT groups. (d) Freeze time during the cue and contextual fear conditioning test in the four groups. (e) Swimming speed, Platform+Edge frequency, and Lantency period during Morris water maze test in the four groups. ^∗^*P* < 0.05,^∗∗^*P* < 0.01.

**Figure 4:** The protective effects of Notch inhibition on cognitive deficits depended on autophagy. (a) Western blot analysis and shading analysis of Beclin 1, Atg5, LC3I, and LC3II in Control, high-dose Pb exposure, DAPT, and high-dose Pb exposure+DAPT groups. (b) Western blot analysis and shading analysis of mTOR, p-mTOR, P70s6k, and p-P70s6k in the four groups. ^∗^*P* < 0.05. ^∗∗^*P* < 0.01.

**Figure 5:** Pb exposure induced a low inflammatory response in the gut and gut dysbiosis in mice. (a) Western blot analysis and shading analysis of gut barrier markers, including E-cadherin, Claudin-3, Claudin-1, ZO-2, and ZO-1 in control and high-dose Pb exposure groups. (b) Representative images of hematoxylin and eosin-stained colon sections from control and high dose Pb exposure groups. (c) Representative images of HE stained jejunum sections from control and high dose Pb exposure groups. (d) Shannon diversity index of gut microbiota in the three groups. (e) PCOA analysis of gut microbiota in the three groups. ^∗^*P* < 0.05.^∗∗^*P* < 0.01.

RETRACTED

**Figure 6:** Pb-exposure induced gut dysbiosis are tightly associated with cognitive deficits in mice. (a) Network analysis at the genus level. V: number of nodes. E: number of edges. (b) Gut bacteria with different abundances. (c) Lefse analysis of the three groups. (d) Relationship of bacteria with different abundances. (e) Heatmap of Spearman's rank correlation coefficients between serum lead, freeze time in context, freeze time in conditioning stimulus, and gut bacteria abundance. *n* = 8 in control, *n* = 9 in low dose Pb exposure group, and *n* = 8 in low dose Pb exposure group. ^∗^*P* < 0.05.^∗∗^*P* < 0.01.

## Data Availability

A detailed analysis of the data is provided to support the conclusions made in this article.
